RETRACTED

# Chemopreventive Efficacy of *Andrographis paniculata* on Azoxymethane-Induced Aberrant Colon Crypt Foci *In Vivo*

**DOI:** 10.1371/journal.pone.0111118

**Published:** 2014-11-12

**Authors:** Nawal Al-Henhena, Rozaida Poh Yuen Ying, Salmah Ismail, Wala Najm, Shaden A. M. Khalifa, Hesham El-Seedi, Mahmood Ameen Abdulla

**Affiliations:** 1 Department of Biomedical Science, Faculty of Medicine, University of Malaya, 50603 Kuala Lumpur, Malaysia; 2 Department of Experimental Hematology, Karolinska University Hospital, SE-141 86 Stockholm, Sweden; 3 Division of Pharmacognosy, Department of Medicinal Chemistry, Uppsala University, Box 574, SE-75 123, Uppsala, Sweden; 4 Institute of Biological Science, Faculty of Science, University of Malaya, 50603 Kuala Lumpur, Malaysia; Rutgers University, United States of America

## Abstract

*Andrographis paniculata* is a grass-shaped medicinal herb, traditionally used in Southeast Asia. The aim of this study was to evaluate the chemoprotective effects of *A. paniculata* on colorectal cancer. *A. paniculata* ethanol extract was tested on azoxymethane (AOM)-induced aberrant crypt foci (ACF) *in vivo* and *in vitro*. *A. paniculata* treated groups showed a significant reduction in the number of ACF of the treated rats. Microscopically, ACF showed remarkably elongated and stratified cells, and depletion of the submucosal glands of AOM group compared to the treated groups. Histologically, staining showed slightly elevated masses above the surrounding mucosa with oval or slit-like orifices. Immunohistochemically, expression of proliferating cell nuclear antigen (PCNA) and β-catenin protein were down-regulated in the *A. paniculata* treated groups compared to the AOM group. When colon tissue was homogenized, malondialdehyde (MDA) and nitric oxide (NO) levels were significantly decreased, whereas superoxide dismutase (SOD) activity was increased in the treated groups compared to the AOM group. *A. paniculata* ethanol extract showed antioxidant and free radical scavenging activity, as elucidated by the measure of oxidative stress markers. Further, the active fractions were assessed against cell lines of CCD841 and HT29 colon cancer cells.

## Introduction

Colorectal cancer continues to afflict several thousands of males and females per year, accounting for about 10% of cancer-related deaths and weighed as the third commonest malignancy in Malaysia as reported in 2007 [1]. Therapeutic modalities such as chemotherapy and radical colostomy are considered curative for localized manageable cases, in fact they are acknowledged for the noticed increase in the five-year survival [2]. The fluoropyrimidine 5-fluorouracil (5-FU) is an anti-tumour agent widely used in the treatment of solid tumours, including colorectal cancers [3]. It is the most potent agent that can be used solely for colorectal cancer treatment in an advanced stage [4]. Fluorouracil is one of the chemotherapeutic drugs of choice for the treatment of colon, rectum, stomach, and pancreatic tumours and is also regularly used to alleviate breast benign and malignant lumps. Unfortunately, fluorouracil among other chemotherapies has side effects, which include diarrhoea, heartburn and sores in mouth and on lips. Approximately 20% of the patients develop symptomatic organ failures, manifested as stomach cramps, painful urination, and difficulty in breathing accompanied by fever or chills. The complications of the standard chemotherapies were attributed to their nature as antimetabolites that impair the production of the essential proteins followed by secondary cellular degradation. The strong impact of the fluorouracil on the body tissues increases the risk for delayed unwanted consequences. However, cessation of fluorouracil therapy is not always a choice, because the symptoms of the polyp formation and carcinogenic early/late stage affect the patient's quality of life even more. Currently, a great number of natural products have been found possessing anti-carcinogenic property by counteracting different etiological factors [5]. Habitual consumption of medicinal plants are known to improve mitochondrial bioenergetics and inhibit various secondary sources of reactive oxygen species (ROS), thus reducing the risk for carcinogenesis [6]. Studying specific natural product molecules selected on the basis of the inhibition of multiple processes responsible for the production of proinflammatory mediators and stimulating the transcriptional machinery necessary for mitochondrial biosynthesis may be a feasible approach for the prevention and treatment of numerous types of cancer.

RETRACTED

*Andrographis paniculata* is a potential cure for several malignancies [7] and treatment of several non-malignant disorders functioning as anti-diabetic [8], anti-ulcerative [9], anti-bacterial and anti-fungal [10], antioxidant [11], anti- HIV [12], antioedema and analgesic [13], anti-inflammatory [14], wound healing [15] renal-protective [8], cardio-protective and hepato-protective [16] agent. An increase in plasma concentration of andrographolide (AP) and 14-deoxy-11, 12-didehydroandrographolide (DIAP) were observed from 30 min to 3 hours after oral administration of the *A. paniculata* extract [17].

Today, a combination therapy of *A. paniculata* and *Elutherococcus senticosus* is commonly used in traditional Chinese medicine [18]. *A. paniculata* (Burm.f.) Nees, known as Kalmegh or “King of Bitters” is a common grass-like species, genus Andrographis (family Acanthaceae). It is indigenous to the Southeast Asian countries (e.g., China and India). It has been documented before 2500 BC in the ancient Ayurvedic system of healthcare and longevity [19]. It is also popular in Chinese medicine, and was recently approved as an anti-influenza remedy in Scandinavia [20]. Both fresh and dried *A. paniculata* leaves, as well as the juice extract, are widely endorsed in folk medicines as a curative lead for liver disorders, bowel and colic pain, general debility, and convalescence after fevers [21]. *A. paniculata* is currently being used as a substitute for chemotherapeutic agents such as fluorouracil to avoid serious side effects for long-term survivors. Although clinical results of *A. paniculata* are constantly improving, the mechanisms of the early events in the prevention of colorectal cancer formation have not yet been satisfactorily elucidated. In this study we wanted to examine the effect of *A. paniculata* against azoxymethane (AOM)-induced aberrant crypt foci (ACF) in colon.

Experimentally, AOM is a standard carcinogen that is usually used to induce colon cancer *in vivo*. AOM has proven to be useful in the chemopreventive screening of dietary supplements such as indigestible sugars, red meat, and green tea [22]. To examine the mechanisms involved in the colorectal carcinogen associated with AOM induction, Sprague Dawley rats were used for testing the anti-oxidative and anti-proliferative influence of *A. paniculata* ethanol extract and its corresponding fractions. In this report, AOM was administered twice over a time span of two weeks to develop cryptal foci that mimic the features of early colorectal carcinogenic lesion. Application of AOM exhibited various histopathological, biochemical and immunohistochemical alterations of colorectal adenoma precursors. Our observations throughout the two weeks of injection and eight weeks following up of experimental course reflect the effects of *A. paniculata* treatment.

Further, the rat colorectal model of ACF was developed in our group as part of our on-going investigations to examine the biological implication of natural products from medicinal plants versus synthetic compounds in the *in vivo* situation. Accumulating body of data recognised ACF as benign adenomatous polyps that progress into an advanced adenoma with high-grade dysplasia that later can lead to an invasive cancer [23]. The development of cryptal foci in the colon is generally accepted as precancerous lesions. The dosage of *A. paniculata* extracts and fractions were adjusted to simulate the effects of fluorouracil regimen used in practice. In total, this study and our future investigation goal will be to shed light on the mechanism underlying the prevention of colon cancer and the development of safer alternatives in order to enhance prophylactic treatment strategies and/or optimize the current regimen by adding complementary natural products.

RETRACTED

## Material and Methods

### Plant material

*A. paniculata* was obtained from Ethno Resources Sdn. Bhd., Selangor, Malaysia and identified at the Herbarium of Rimba Ilmu, Institute of Biological Science, University of Malaya, Kuala Lumpur. The plant was washed, dried, and grounded. The ethanol extract was obtained by soaking 100 g of the powdered plant in 1000 ml of 95% ethanol at room temperature for 3–4 days. This was followed by evaporation under low pressure at 45°C to obtain the crude ethanolic extract. The final yield was 8.7 mg crude extract for every 100 mg plant material. The crude extract was stored at −20°C until further use.

### Experimental animals

Healthy adult female SD rats (6–8 weeks old, between 150–180 g) were placed in individual cages at the Animal House, Faculty of Medicine, University of Malaya. This study was conducted on rats because of the ease in handling, injecting, and feeding these rats. In addition, the processing of blood samples and organs of rats was easier compared to those of mice. The study was approved by the Ethics Committee for Animal Experimentation, Faculty of Medicine, University of Malaya, Malaysia [Ethic No PM/07/05/2011/MMA (a) (R)]. Thirty rats were equally divided into five groups within this study. Group 1 (normal group) was injected subcutaneously with normal saline once a week for two weeks and fed orally with 10% Tween 20 for two months. Group 2 (AOM control group), Group 3 (FU treated group), Groups 4 (*A. paniculata* treated groups) and group 5 (*A. paniculata* sub-lethal treated groups) were injected subcutaneously, each with 15 mg/kg AOM once a week for two weeks, and continued to be fed, orally with 10% Tween 20 (daily), intra-peritoneal injection with fluorouracil (5-FU) 35 mg/kg twice a week for a month, and the oral administration of *A. paniculata* plant extract was scheduled at two doses of 250 mg/kg and 500 mg/kg (daily), respectively.

For the acute toxicity study, one dosage level was chosen in such a way that the dose was ten times the low dose of chemopreventive study (2500 mg/kg).

### Chemicals

Azoxymethane (AOM; Sigma Chemical Co., St. Louis, MO, USA) was dissolved in 0.9% normal saline and administered subcutaneously at a dosage of 15 mg/kg body weight once a week for 2 weeks, to induce ACF in colon [24]. The reference drug, fluorouracil (5-FU; Sigma Chemical Co., St. Louis, MO, USA), was dissolved in 0.9% normal saline and administered intraperitoneally at a dosage of 35 mg/kg body weight twice a week in accordance with a previously described protocol [25].

RETRACTED

### Column chromatography

Column chromatography was performed to fractionate the plant extract [26] by a Kontes glass cylinder column (2.0×50 cm glass column) containing packed silica gel 60 (0.063–0.200 mm, 70–230 mesh (Merck, Germany)). Starting from the lowest to the highest polarity, different concentrations of eluting solvents (hexane, ethyl acetate, methanol, acetone, acetonitrile, and water) were passed through the column (1 g of the plant extract per 5 ml solvent was used). The eluted fractions were collected.

### Thin layer chromatography (TLC)

The eluted fractions were analyzed via thin layer chromatography using aluminium foils precoated with silica 60 F254 plate (20 cm ×20 cm width and 0.2 thickness) (Merck, Darmstadt, Germany). The TLC analysis was performed using a mixture of ethyl acetate and ethanol. After UV light visualization at 240 nm and 360 nm, the similar collected fractions were combined to obtain the main fractions of the extract depending on the similarities of retention factor and spot colours. Six major fractions (ANF1, ANF2, ANF3, ANF4, ANF5, and ANF6) were obtained. The chemopreventive effects of the fractions were assessed in vitro against human colorectal adenocarcinoma cell line HT29 and cytotoxicity for human colon epithelial cell line CCD 841.

### Liquid chromatography/mass spectrometry (LC/MS)

The fractions that showed positive results were further identified by HPLC and LC-MS. The Agilent 1200 Series HPLC system with capillary pump and degasser, micro well plate sampler with thermostat, and agilent 6520 accurate-mass Q-TOF mass spectrometer with dual ESI source was used. The Agilent Zorbax SB-C18 (0.5×150 mm, 5 µm) with the following conditions: Part no - 5064–8256; flow rate −18 µL/min from agilent 1200 series capillary pump (micro flow); injection volume: 1 uL; positive polarity −0.1% formic acid in water (solvent A); and 90% acetonitrile in water with 0.1% formic acid (solvent B) was employed. Analysis was performed by negative polarity 5 mM ammonium formate in water (solvent A) and 90% acetonitrile in water with 5 mM ammonium format (solvent B). Sample analysis was performed with the following elution gradients: 0 min −3% (B) in (A); 30 min −100% (B) in (A); 38 min −100% (B) in (A); 38.1 min −3% (B) in (A); and 46 min −0% (B) in (A).

### The 2, 2-diphenyl-1-picryl-hydrazyl (DPPH) assay

Determination of the free radical scavenging activity of the plant extract was established spectrophotometrically using DPPH. DPPH is originally violet, which changes to yellow upon interaction with the antioxidants [27]. The DPPH working solution was prepared using 95% ethanol in a concentration of 3.94 mg/100 ml. The sample and the DPPH reagent were mixed well and incubated for 20 min at room temperature in a dark place. The absorbance was measured at 517 nm in triplicates. Vitamin C was used as a standard indicator following the protocol of Ikram [29]. The activity of the extract was calculated based on the percentage of scavenged DPPH.

RETRACTED

### Total phenolic and total flavonoid contents

Total phenolic content (TPC) was determined based on the Folin-Ciocalteu spectrophotometric method with slight modifications. The measurement was compared to a standard curve of gallic acid (GA) solution and the value was expressed as milligrams of GA equivalents (GAE) per gram of the plant extract (mg GAE/g db) [29]. Total flavonoid (TF) content was measured using the aluminum chloride colorimetric method. The measurement was expressed as quercetin equivalents in mg (QE)/g of the extract [30]. The assays were carried out in triplicates.

### Ferric-reducing antioxidant potential (FRAP) assay

Ferric-reducing antioxidant potential (FRAP) assay was performed as described by Benzie and Strain [31]. The FRAP reagent was prepared by mixing 16.7 mMFeCl_4_.6H_2_O and 8.3 mM 2,4,6-tripyridyl- s-triazine (TPTZ) with 250 mM acetate buffer, pH 3.6. The ethanol extract was added to the freshly prepared FRAP reagent in a 96-well plate. The antioxidant potential of the plant extract was calculated using FeSO_4._7H_2_O as a standard at 400–1000 mM and the absorbance was read at 0 and 4 min at 593 nm. Vitamin C, gallic acid (GA), butylated hydroxytoluene, and quercetin were used as positive controls [28].

### Nitric oxide (NO) concentration

For the determination of nitric oxide concentration, the stable conversion product of nitric oxide to nitrite (NO_2_) was measured using the Griess reagent as described earlier [32]. A series of dilutions was prepared from a 1 mg/ml stock of the plant extract. At every concentration, 50 µl of the extract was transferred into 96-well microplates and an equal volume of sodium nitroprusside was added. The preparation was incubated for 1 h under visible polychromatic light (light and heat). Griess reagent (100 µl) was then added to the mixture at room temperature. The percentage inhibition was obtained by calculating the ability of the plant extracts to inhibit nitric oxide formation compared to the control (vitamin C), which was set at zero percent inhibition [33]. The absorbance was read at 550 nm using sodium nitrite as a standard [34]. Percentage inhibition was defined as [(Ao – As)/Ao)]*100, where Ao is the absorbance of control and As is the absorbance of test samples.

RETRACTED

### Toxicity test

The acute toxicity study was performed preliminarily to determine the safe dosage of *A. paniculata*. For this purpose, sixteen healthy rats were divided randomly into two groups. The two groups were vehicled either with10% Tween 20 or 2500 mg/kg plant extract, respectively. The rats were deprived of food and water one night before the administration. After vehicling, water and food was further withheld for 3–4 h. The rats were initially observed for 30 min; then the observation continued for 2, 4, 24 and 48 h. The appearance of clinical or toxicological symptoms of mortality over a period of two weeks was recorded and the body weights of the two groups were measured weekly. All rats were sacrificed with overdose of anaesthesia consisting of ketamine and xylazine at 50 and 5 mg/kg body weight, respectively. Biochemical and histological (liver and kidney) parameters were evaluated according to the standard methods of Organization for Economic Co-operation and Development (OECD) [35]. Additionally, the colon, liver and spleen weights of all groups were measured after the rats were sacrificed.

### ACF counting

All rats were sacrificed by cervical dislocation at the end of the experimental ten weeks under a combined overdose of ketamine and xylazine at 50 and 5 mg/kg body weight, respectively. Colons of the sacrificed rats were removed and washed with cold phosphate buffered saline (PBS). Colons were dissected longitudinally and each colon was cut evenly into three segments (proximal, middle, and distal). The colon segments were fixed in 10% formalin for 5–10 min, and stained with methylene blue (0.2% in PBS solution) for 15–20 min in order to visualize the crypts [36]. The colon segments were placed on inverted microscope with the intestinal mucosa facing up and the number of the crypts foci was counted on random observational fields at a magnification of 2X and 4X.

### Histopathological examination

Colon tissue was sectioned using a programmed tissue-processing machine, after which the 5 µm thick sections were embedded in paraffin wax. The liver and kidney of normal and treated groups were also histologically tested to determine the histolopathological changes that occurred in response to the long-time of plant oral administration. The sections were stained with hematoxylin and eosin for histological and immunohistochemical evaluation.

### Immunohistochemical staining

Five µm thick colon sections were mounted on slides coated with poly-lysine then dried overnight in an oven at 50°C. Sections were deparaffinised and rehydrated in graded alcohols. For the retrieval of antigen target, a 10 mM sodium citrate buffer solution was used. The tissue was then rinsed in PBS prior to immunohistochemical staining. Immunohistochemical procedures were done according to the manufacturer's protocol (Dako ARK USA) where the proliferating cell nuclear antigen (PCNA) and β-catenin proteins are an indicator of proliferative alterations and the avidin biotin and peroxidase reactions served as the fluorescent markers. Negative control sections were processed similarly, but with the omission of the primary antibodies. All sections were viewed under a light microscope (100X magnification).

RETRACTED

### Biochemical parameters

Biochemical parameters were performed using the standard automated analyser at the Central Diagnostic Laboratory, University of Malaya Medical Centre. Blood samples were collected in gel activating tubes and centrifuged at 3000 rpm for 10 min. The serum was separated and calibrated for the presence of creatinine, total protein, albumin and glucose levels, as well as alkaline phosphatase (ALP), alanine aminotransferase (ALT), aspartate aminotransferase (AST) and lactate dehydrogenase (LDH).

### Antioxidant activity in colon homogenate

The colon tissue was rinsed with ice-cold PBS solution, pH 7.4 to remove extra cells or debris. Protease (a mixture of protease enzymes used for the inhibition of serine, cysteine, aspartic proteases and amino peptidases) was employed to break the cellular interstitial layer. One gram of colon tissue was homogenized in 5–10 ml of cold buffer, and centrifuged at 4500 rpm for 15 min at 4°C. The tissue homogenate supernatant was used for the observation of superoxide dismutase (SOD) activity. Thiobarbituric acid reactive substances (TBARS) assay were used to measure malondialdehyde (MDA) for lipid peroxidation levels and nitric oxide (NO) levels. All measurements were performed using commercial kits (Cayman Chemical Company, U.S.A).

### *In vitro* chemopreventive assessment

The human epithelial colon cell line CCD 841 (ATCC CRL-1790) and colorectal adenocarcinoma cell line HT29 (ATCC HTB-38) was a gift from Department of Molecular Medicine, Faculty of Medicine University of Malaya. They were grown in RPMI medium supplemented with 10% (v/v) foetal bovine serum (FBS) and 1% antibiotic (penicillin and streptomycin), and were incubated at 37°C in a humidified incubator with 5% CO_2_. The cells were sub-cultured periodically to keep them in an exponential growth phase. The CCD 841 and HT29 cells were seeded in 96-well plates at the density of 5×10^5^ viable cells/well. Both cell types were exposed to different concentrations of plant extract and its fractions (6 fractions), and were incubated for 24–48 h to allow cell adherence. Then, 10 µl MTT (5 gm/ml PBS) was added to each well and re-incubated for 4 h. The medium containing MTT was removed and 100 µl DMSO was added. The absorbance was read at 595 nm using the microplate reader and cell viability was calculated.

RETRACTED

### Statistical analysis

The counts from different treatment groups were calculated from numerous observational fields and analysed for each individual experiment (n). Each experiment was repeated at least 3 times and triplicate samples were counted for each condition. Recorded data were fed into a computer program (Window XP, Excel). One-way ANOVA for independent samples was performed followed by Tukey's post-hoc test using SPSS version 19 (SPSS Inc. Chicago, IL, USA). A value of P<0.05 was considered significant and all values were reported as mean ± SD.

## Revised Results

### Acute toxicity

No mortalities were observed in the treated animal groups. In addition, there were no visible manifestations of hepatotoxic and nephrotoxic effects, at sub-lethal doses. Furthermore, the blood biochemistry and histopathology demonstrated no major destruction of the affected tissues neither in the treated groups nor the control. Thus, drug related toxicity was not detected even at the highest dose investigated (2500 mg/kg in this case) and throughout the observational course of 14 days. The sub-lethal dose was previously recommended by OECD [35].

### Body, colon, liver, spleen and kidney weights and histological changes of liver and kidney

In terms of body weight, rats treated with the ethanolic extract were heavier compared to the AOM control group, whereas rats treated with 5-FU were lighter (Table 1). The local effect of the treatments on the organs was tested and it was found that the colon weights was higher in respect to the AOM control group with no major differences in liver, spleen and kidney weights between the groups. The long term oral administration of *A. paniculata* revealed no histopathological changes of liver and kidney in plant treated groups with respect to the normal (vehicle) group (Figure 1).

**Figure 1:** The histological changes of major organs (Kidney and Liver) in *A. paniculata*-treated AOM-induced cancer. They showed normal and no related toxicity in liver and kidney tissues as they are the main organs for detoxification process in the body.

**Table 1:** Effect of *A.paniculata* on weights of body, liver, colon, spleen and kidney.

Group/Weight	Body (gm)	Colon (gm)	Liver (gm)	Spleen (gm)	Kidney (gm)
Normal group	307.33±12.65	2.62±0.05	8.16±0.23	0.88±0.05	2.51±0.15
AOM control group	314.50±19.56	3.14±0.24	9.87±0.67	0.86±0.05	2.82±0.36
FU group (AOM +5-FU35 mg/kg)	383.50±17.38	2.18±0.16	10.09±0.05	0.66±0.03	2.93±0.07
AOM +*A. paniculata* 250 mg	426.67±28.48*	4.08±0.32*	12.04±0.93	0.86±0.04	2.79±0.31
AOM +*A. paniculata* 500 mg	419.33±13.48*	4.11±0.35*	12.51±0.66	1.0±0.07	2.70±0.27

Values expressed as mean ± S.E.M. *Significant at the 0.05 level.5-FU: 5-Fluorouracil; AOM: azoxymethane.

RETRACTED

### Aberrant crypt foci number in rats colons

Rats were sacrificed and the colons were observed and scored for ACF count (Table 2). No ACF formation was observed in the control group not exposed to AOM. The treated rats had a lower ACF count, with respect to the AOM control rats (p<0.01). Additionally, the distribution of ACF in colon was different in various colon segments. ACF were mainly found in the middle and distal parts of colon in extract-treated groups, whereas ACF were mainly found in the middle and proximal parts of the colon in the AOM control group and FU-treated group. The treated rats showed a significant reduction in the number of ACF in each colon segment. In total, the extract treatment significantly reduced the number of crypts per focus (Table 3).

**Table 2:** Effect of *A. paniculata* on AOM-induced ACF in rat colon.

Group	ACF	ACF distribution at the colon segments		
	Total	Proximal	Middle	Distal
AOM control group (AOM 15 mg/kg)	150±21.01	36.8±4.60	83±14.5	30±9
FU group (AOM+5-FU35 mg/kg)	41±9.68**	5±1.2**	32±9.74**	3.6±1.7**
AOM +*A. paniculata* (250 mg/kg)	49±5.78**	7±0.88**	15.6±1.0**	26±7.06**
AOM +*A. paniculata* (500 mg/kg)	38±4.17**	8.6±1.6**	16.6±2.1**	13±2.1**

All values are expressed as mean ± S.E.M. **Significant difference at p<0.01. 5-FU: 5-fluorouracil; ACF: aberrant crypt foci; AOM: azoxymethane.

**Table 3:** Effects of *A. paniculata* on the numbers of crypts per focus in AOM-induced ACF in rat colon.

Group	Number of foci containing:				
	1 crypt	2 crypts	3 crypts	4 crypts	≥5 crypts
AOM control group (AOM)	26±7.15	36±8.37	31±4.4	25±1.4	30.8±7.3
FU group (AOM +5-FU)	10±2.1**	9±2.3**	9±2.6**	5±1.5**	8±2.6**
AOM +*A. paniculata* 250 mg/kg	6±2.8**	11±1.7**	15±3.1**	9±2.06**	7±1.5**
AOM +*A. paniculata* 500 mg/kg	4±1.0**	11±0**	11±2.0**	9.6±1.4**	6±1.3**

All values are in mean ± S.E.M. **Significant difference at p<0.01 (ANOVA, Tukey's post hoc).

5-FU: 5-Fluorouracil; AOM: azoxymethane.

### Blood biochemical parameters

Lactate dehydrogenase (LHD) was significantly lower in treated groups compared to AOM group (p<0.05) (Table 4). However there was no difference in the level of urea, creatinine, total protein, albumin, glucose, and enzymes (ALT, AST, ALP) (p>0.05).

**Table 4:** Effect of *A. paniculata* on biochemical parameters.

Dose	Total protein (g/L)	Albumin (g/L)	Glucose (mmol/L)	Creatinine (umol/L)	ALP (IU/L)	ALT (IU/L)	AST (IU/L)	LDH* (U/L)
Normal group	63.83±0.49	9.83±0.31	7.20±0.82	29.33±3.84	110.67±9.92	47.17±4.1	199.0±12.16	1373.67±137.29
AOM control group	63.67±0.65	12.8±0.41	8.73±0.25	43.67±3.75	110.67±8.8	51.0±2.15	178.5±9.4	1823.50±97.96
FU treated group	65.67±1.5	12.16±0.17	7.20±0.45	46.0±1.32	133.17±7.2	52.3±2.78	164.83±10.88	776.33±47.32*
(250 mg/kg).*A. Paniculata*	68.0+1.54	13.67±0.42	9.52±0.99	41.167±3.28	117.67±11.02	87.83±14.56	186.42±23.4	646.67±68.52*
(500 mg/kg).*A. Paniculata*	68.167±1.49	13.5±0.62	9.64±0.53	33.3±1.3	118.17±15.66	57.0±2.4	133.0±12.68	682.33±102.42*

All values are in mean ± S.E.M. **Significant difference at p<0.01 (ANOVA, Tukey's post hoc).

5-FU: 5-Fluorouracil; AOM: azoxymethane. Alkaline phosphatase (ALP), alanine aminotransferase (ALT), aspartate aminotransferase (AST) lactate dehydrogenase (LDH).

RETRACTED

### Malondialdehyde, nitric oxide and superoxide dismutase bioassays in colon homogenate

Malondialdehyde (MDA), nitric oxide (NO) levels and superoxide dismutase (SOD) activity of the colon homogenate differed among groups. Malondialdehyde levels were significantly lower in *A. paniculata* (4.7±0.33, 4.1±0.46 at 250 mg/kg, 500 mg/kg, respectively) and FU treated rats (3.6±0.12 µm) (Figure 2). Likewise, nitric oxide levels were significantly lower in *A. paniculata* treated rats with a value of 10.9±0.32 µm at 250 mg/kg and 8.2±1.7 µm at 500 mg/kg (Figure 2). Moreover, SOD activity showed values of 11.5±0.9 and 11.1±0.2 U/ml at dosages of 250 and 500 mg/kg (Figure 2).

**Figure 2:** Effect of *A. paniculata* on superoxide dismutase (SOD) activity, malonaldehyde (MDA) level and nitric oxide (NO) level in AOM induced tissue. All values are represented as mean ± SEM. Significant difference at *P<0.01, ** P<0.001(ANOVA, Tukey's). FU: Fluorouracil; AOM: azoxymethane.

### DPPH, FRAP, and NO bioassay

Antioxidant activity was evaluated based on the free radical scavenging activity of the samples using the 2, 2-diphenyl-1-picrylhydrazyl (DPPH) free radical scavenging assay. *A. paniculata* ethanol extract showed a remarkable activity with BHT, with an IC50 value of 57.08 µmol (Table 5). Furthermore, the ferric reducing antioxidant potential (FRAP) assay to confirm the above results by measuring the reduction of iron from the ferric form (Fe3+) to the ferrous form (Fe2+). The ability of the extract to reduce Fe3+ to Fe2+, was 4676.2±0.07, mimicking those of BHT, at 5228.6±0.01 (Table 5). Nitric oxide (NO) radical scavenging activity (172.9%) was comparable to vitamin C at 183.7%. The nitric oxide radical scavenging activity was utilized to evaluate the power of the plant extract to scavenge free radicals in vitro.

RETRACTED

**Table 5:** Antioxidant activity of *A. paniculata* in vitro.

	DPPH(IC50 µmol/L)	FRAP (mmol/g)	TPC (mg/g)	TF (mg/g)	Nitric oxide%
BHT	8.06±0.28	5228.6±0.01	------	------	------
Vitamin C	------	------	------	------	183.7±0.89
Gallic acid	------	------	1015.3±0.004	------	------
Quercetin	------	------	------	775.71±0.009	------
*A. paniculata*	57.08±1.04	4676.2±0.07	242.67±0.007	142.86±0.005	172.9±0.85

Values represent mean ± SEM for triplicates; BHT-butylated hydroxytoluene.

### Total flavonoids and phenolic contents

Total phenolic and flavonoid contents (TPC and TFC, respectively) were assessed for the plant extract. TPCs of the extract were 242.67±0.007 mg, expressed as gallic acid equivalent in mg per g of the plant extract. TFC levels were 142.86±0.005, expressed as quercetin equivalents in mg per g of the plant extract (Table 5).

### Histopathological study using haematoxylin and eosin stain

The histological features of colon cells were observed by haematoxylin and eosin (H&E) staining. Histological examination of AOM colon tissue showed remarkably elongated and slightly stratified cells. Additionally, the AOM colon tissue showed proliferating mucosal glands and shrinkage of submucosal layer with marks of mucin depletion. The morphological and histological alterations represent early stages of cancer transformation (Figure 3).

**Figure 3:** Cross-section of the rat colon stained with hematoxylin and eosin: (A) Normal group with normal crypts, (B) AOM control group (C) FU treated group, D) 250 mg/kg *A. paniculata* treated group, (E) 500 mg/kg *A. paniculata* treated group (100X magnification). For (B), arrow indicated the elongated and slightly stratified nuclei found in AOM control group, showing depletion of mucin. For (A), (C), (D) and (E) which represented the normal cells, the arrows indicated crypts with round nuclei which are normal.

### Methylene blue staining of ACF

ACF were visualized by staining with 0.2% methylene blue, and was observed predominantly in the middle and distal colon and to a lesser extent in the proximal colon. ACF were slightly elevated above the surrounding mucosa with oval or slit-like orifices (Figure 4). The aberrant crypts had irregular luminal elongated crypts and thicker epithelial lining with decreased goblet cells. The lateral view demonstrated that the ACF protruded towards the lumen.

**Figure 4:** Effect of *A. paniculata* on ACF count: (A) Normal group with normal crypts, (B) AOM control group (ACF with multiple crypts> five), (C) FU treated group, (D) 250 mg/kg *A. paniculata* treated group, (E) 500 mg/kg *A. paniculata* treated group (methylene blue staining. (4X magnification). The arrows indicated the crypts that were more than five foci in AOM control group and less than five foci in all treated groups.

RETRACTED

### Immunohistochemical staining

AOM group had high expressions of PCNA and β-catenin proteins (Figures 5, 6) compared to the other three groups based on the immunohistochemical appearance. The sections of the AOM group showed the brownish positive colour revealing the up-regulation of PCNA protein, in contrast to the treated groups where the bluish appearance indicated PCNA protein down-regulation. Overexpression of beta catenin protein in AOM control group was observed with respect to treated groups.

**Figure 5:** (**a**): Regulation of PCNA in the colon tissue of rats (A) Normal group (B) AOM control group (C) FU treated group, (D) 250 mg/kg *A. paniculata* treated group, and (E) 500 mg/kg *A. paniculata* treated group (100X magnification). (**b**): Regulation of PCNA protein expression in the colon tissue of normal and AOM induced rats. All values are in mean ± SEM. FU: Fluorouracil; AOM: azoxymethane.

**Figure 6:** Regulation of β-catenin in the colon tissue of rats. (A) Normal group (B) AOM control group (C) FU treated group, (D) 250 mg/kg *A. paniculata* treated group, and (E) 500 mg/kg *A. paniculata* treated group (100X magnification). In the AOM and treated groups the arrows indicated to the cells expressed the β-catenin protein. The β-catenin showed to be more expressed in AOM control group than that of treated groups.

### Chromatographic profiling of A. paniculata

The crude extract was separated by column chromatography into six fractions, according to the differences in molecular size and polarities. Their anti-proliferative effects were investigated against HT29 and CCD-841. High inhibition was obtained with fractions 4 and 5 (ANF4 and ANF5) (Figure S1) and moderate inhibition with fractions 1 and 2 (ANF1 and ANF2). The cell viability decreased to 3.53% and 6.10%, at concentrations of 50 µg of ANF4 and ANF5, respectively. In contrast, low inhibition was observed in the CCD-841 colon cells with ANF4 and ANF5. At the same concentration, the cell viability was detected at 58.74% and 55.8%, respectively. ANF5 was studied further by LC-MS to identify the active compounds and eight peaks were distinguished (Figure 7). The isolated compounds (Table 6) were characterized and mainly diterpenoids were evident. Diterpenoids in the fractions included andrographolide, 14-deoxyandrographolide, and 14-deoxy-11, 12-didehydroandrographolide in addition to amentoflavone and epicatechin.

**Figure 7:** (**a**): Chromatogram (a & b) of *A. paniculata* in negative mode (in 10% acetonitrile in water +0.1% formic acid). Peaks 1 & 2 represented the (14-deoxy-11, 12-didehydroandrographolide) and (Amentoflavone) compounds. (**b**): Chromatogram (a & b) of *A. paniculata* positive mode (in 10% acetonitrile in water +0.1% formic acid). The highest peak (5) represented the main fraction compound (Andrographolide).

RETRACTED

**Table 6:** Identification of the main components of A. paniculata F5 by LC-MS positive and negative modes.

No. of Peaks	Rt	Formula	Mass	m/z	Polarity	Compound
1	14.8	C_20_ H_28_ O_4_	332.2	331.19	Negative	14-deoxy-11, 12-didehydroandrographolide
2	14.89	C_30_ H_18_ O_10_	542.272	542.266	Negative	Amentoflavone
3	12.4	C_20_ H_28_ O_4_	332.2	665.403	Positive	14-deoxyandrographolide
5	14.8	C_20_ H_30_ O_5_	350.22	701.43	Positive	Andrographolide
8	20.95	C_15_ H_14_ O_6_	290.268	290.268	Positive	Epicatechin

## Discussion

Colorectal epithelial homeostasis is attributed to the balance between cell proliferation and cell death. Colorectal cancer arises from abnormal growth of the colon cells with excessive proliferation [37]–[38]. Oxidative stress plays an important role in the molecular mechanism of colon cancer development and progression [39]. Many studies have shown that a diet rich in phytochemicals is associated with reduction in the risk of cancer [40]. The wide range of chemical compounds that are present in natural dietary products has been approved as antioxidant and chemopreventive entities [41]. *A. paniculata* is known to be a rich source of many bioactive compounds with a broad range of pharmaceutical effects [42]. Extracts of *A. paniculata* were found to inhibit the formation of oxygen derived free radicals [43]. Some of the plant bioactive compounds of these extracts belong to the diterpenoid and flavonoid classes [42]. Dietary phytochemicals and herbs similar to *A. paniculata*, especially its polyphenolic components have the potential in the prevention of colon cancer [44].

AOM induction regimen has been reported to cause aberrant crypt foci in the colon, which was confirmed in our present study by the observation of crypt formation and mucosal damage [45]. However, the crypt formation could not be caused solely by inflammation due to the AOM injection, hence neither inflammatory cells nor elevation in inflammatory cytokines/blood parameters were observed. The higher expression of antioxidant modulators may be a result of a protective mechanism following both tissue injury and inflammation [46]. The uptake of the free radicals could be attributed to the antioxidant scavenger potential of *A. paniculata* as confirmed by DPPH, NO, and FRAP bioassays [47]. Recently reported the effects of some medicinal plants as chemopreventive agents against colon cancer. We report that *A. paniculata* specifically affected the number and features of the cryptal foci. The resistant small-sized crypts showed minor signs of mucosal elongation and stratification: minimal shrinkage of the submucosal layer with no obvious depletion of intestinal glands. This structure and mechanical resistance significantly influenced the number and distribution of the foci along the three main segments of the colon.

RETRACTED

Our *in vitro* examinations have shown that the colon homogenate of *A. paniculata* treated animals had a lower level of MDA than control. Since the colon homogenate was obtained from defined colon segments, we consider the parameter changes to reflect a remodeling of colon oxidative stress based on reduction of lipid peroxidation. This was in agreement with our observation of the dramatic decline of serum LDH rather than other biochemical markers such as creatinine, TP, Glu, Alb, ALP, ALT, and AST. LDH is considered a prognostic marker in malignancies and in particular for colorectal cancer [48]. β-catenin is one of the specific genes and a dual function protein, regulating the coordination of cell–cell adhesion and gene transcription. Mutations and overexpression of β-catenin are associated with many cancers, including colorectal carcinoma. The accumulation of functionally altered beta catenin protein was observed as a consequence of destruction of the adenomatous polyposis, in agreement with several studies [49]–[50]. Another interesting observation was how the cancer colon cells *in vitro* had a significant ability to rapidly adapt to alterations in oxidative stress and respond to the anti-oxidant effect of *A. paniculata* on a time scale of days to weeks. It is therefore likely that the free radical scavenging was increased possibly via high metabolic rate and endothelial NO release.

Since increased SOD activity is associated with catalysis of the superoxides into oxygen and hydrogen peroxide in many cancer models [51], the finding that the *A. paniculata* enhanced SOD activity in rat colon model is associated with positive immunohistochemical-staining of PCNA might suggest that the free radical release in oxidative stress is also associated with increased lipid peroxidation. The high antioxidant property of SOD was reported in cases with colon inflammation as for the management of colitis inflammation and the inhibition of endothelial activation [52]–[53]. The changes in the structure of the mucosa were associated with irregular luminal elongated crypts in response to endothelial stimulation. A combination of an elevation of the endothelial layer towards the lumen and up-regulation of PCNA expression would lead to major alterations of the colon contractility signalling. These data and the suppression of crypt formation are also consistent with a mechanism where the apoptotic cascade is compensating for proliferation alterations of colorectal mucosa.

RETRACTED

The *in vivo* measurements also clearly showed an increase of the animal weight, which suggests not only healthy animals but the satisfactory nutritional supply under our proposed regimen and specifically the remarkable digestion and absorption pharmacodynamics. Liver and kidney tissues revealed no histopathological changes on long term *A. paniculata* oral administration. Possibly the increased colon weight of the treated animals is related to water retention and dilution of the free radical. It should be noted that the improvement of nutritional values following *A. paniculata* would further indicate promotion of the structural and functional integrity of the colon segments. It is noteworthy that the acute toxicity test did not reveal any histopathological changes in the liver and kidney tissues treated with the plant extracts compared to control.

The findings from this study suggested that *A. paniculata* possesses antioxidant, anti-proliferative and antimetastatic activities and hence, has the potential to offer new anti-cancer therapeutic agent. The bioactivity and bioavailability of *A. paniculata* against cancer was suggested to be due to its diterpenoid and flavonoid contents. Previous studies have discussed the relationship between diterpenoids and cancer prevention [54]. Furthermore, diterpenoids have been tested on HT29, the colon cancer cell line, and have potent effect on the inhibition of HT-29 proliferation [55]–[56]. Flavonoid and diterpenes isolated from *A. paniculata* have been reported for their antioxidant properties and their ability to protect cells from lipid peroxidation [43]. Taken together, our results highlight the chemoprotective attribution of *A. paniculata* on the colon mucosal and submucosal layers and propose some possible components of the early/mid stages of carcinogenic cells proliferation and filtration that could be interrupted efficiently after two weeks of administration, guaranteeing the preservation of the colon integrity and functionality.

## Conclusion

When orally administered to rats, the ethanol extract of *A. paniculata* played a role in the intervention of cancer formation. *A. paniculata* changed the morphological identity of the crypts in the mucosa and showed histological alterations that varied from hyperplasia to dysplasia. The formation of less ACF excludes one of the earlier abnormalities that occur during the colorectal cancer induction. Furthermore, *A. paniculata* interfered with the intermediate biomarker for colon cancer development as evidenced by the various levels of certain oxidative stress markers. This may be due to the antioxidative properties of the extracts as free radical scavengers. In addition, *A. paniculata* regulated the genetic and epigenetic features displaying a chemoprotective effect on the colon cells against a potent carcinogen i.e., AOM as documented on the apoptotic and proliferative levels. The effects were generally comparable to those of rats treated with 5-FU.

RETRACTED

## Supporting Information

Figure S1 Effect of *A. paniculata* fractions ANF4 and ANF5 on the viability of (a & c) HT29 colon cancer cells and (b & d) CCD 841 normal colon cells. Data were expressed as the mean ± SEM for triplicates.
(TIF)
